The article "Characterization of a Cross-Reactive, Immunodominant and HLA-Promiscuous Epitope of Mycobacterium tuberculosis-Specific Major Antigenic Protein PPE68" was published in 2014. Journal: PLoS One.

# Characterization of a Cross-Reactive, Immunodominant and HLA-Promiscuous Epitope of *Mycobacterium tuberculosis*-Specific Major Antigenic Protein PPE68

**DOI:** 10.1371/journal.pone.0103679

**Published:** 2014-08-19

**Authors:** Abu S. Mustafa

**Affiliations:** Department of Microbiology, Faculty of Medicine, Kuwait University, Safat, Kuwait; University of Delhi, India

## Abstract

PPE68 (Rv3873), a major antignic protein encoded by *Mycobacteriun tuberculosis*-specific genomic region of difference (RD)1, is a strong stimulator of peripheral blood mononuclear cells (PBMCs) obtained from tuberculosis patients and *Mycobacterium bovis* bacillus Calmette Guerin (BCG)-vaccianted healthy subjects in T helper (Th)1 cell assays, i.e. antigen-induced proliferation and interferon-gamma (IFN-γ) secretion. To confirm the antigen-specific recognition of PPE68 by T cells in IFN-γ assays, antigen-induced human T-cell lines were established from PBMCs of *M. Bovis* BCG-vaccinated and HLA-heterogeneous healthy subjects and tested with peptide pools of RD1 proteins. The results showed that PPE68 was recognized by antigen-specific T-cell lines from HLA-heteregeneous subjects. To further identify the immunodominant and HLA-promiscuous Th1-1 cell epitopes present in PPE68, 24 synthetic peptides covering the sequence of PPE68 were indivdually analyzed for HLA-DR binding prediction analysis and tested with PBMCs from *M. bovis* BCG-vaccinated and HLA-heterogeuous healthy subjects in IFN-γ assays. The results identified the peptide P9, i.e. aa 121-VLTATNFFGINTIPIALTEMDYFIR-145, as an immunodominant and HLA-DR promiscuous peptide of PPE68. Furthermore, by using deletion peptides, the immunodominant and HLA-DR promiscuous core sequence was mapped to aa 127-FFGINTIPIA-136. Interestingly, the core sequence is present in several PPE proteins of *M. tuberculosis*, and conserved in all sequenced strains/species of *M. tuberculosis* and *M. tuberculosis* complex, and several other pathogenic mycobacterial species, including *M. leprae* and *M. avium-intracellulalae* complex. These results suggest that the peptide aa 121–145 may be exploited as a peptide-based vaccine candidate against tuberculosis and other mycobacterial diseases.

## Introduction

Tuberculosis (TB) is a major infectious diseases problem of world-wide distribution and ranks among the top 10 causes of global mortality. In spite of international efforts to control TB, the most recent estimates available for global epidemiology from the World Health Organization suggest that there were 9.4 million incidence cases and 14 million prevalence cases of active disease and 1.7 million people died of TB in 2009 [1]. The impact of current efforts to reduce the global burden of TB, by means of improved diagnosis and chemotherapy, is less than expected [2]. Therefore, additional preventive efforts, which include the development of new protective vaccines against TB, are essential [2].

Previous studies have shown that interferon-gamma (IFN-γ), a cytokine secreted by T helper (Th)1 cells in large quantities, is a major player in protection against TB [3]–[6]. In addition, mycobacterial antigens/peptides are presented to Th1 cells mostly in association with highly polymorphic human leukocyte antigen (HLA) molecules, in particular HLA-DR [6]–[8]. Thus, to be effective in human populations, which are highly HLA-DR heterogeneous, the antigens/peptides selected as anti-TB vaccine candidates should be recognized by Th1 cells in HLA-DR-non-restricted (promiscuous) manner [9].

The comparative analyses of *M. tuberculosis* genome has shown the presence of several regions of difference (RD) between *M. tuberculosis* and other mycobacteria, particularly when compared with the vaccine strains of *M. bovis* BCG [10]. Among these regions, RD1 appears to be the most important region for Th1-cell stimulation because it contains genes that encode two major antigenic proteins of *M. tuberculosis* (ESAT-6 and CFP10), which were recognized by TB patients and latently infected individuals in IFN-γ assays [11]–[13]. However, the RD1 region has been predicted to contain genes that encode 14 *M. tuberculosis*-specific proteins [14]. By using pools of chemically synthesized peptides corresponding to each RD1 protein, it has been shown that all of these proteins were recognized by Th 1 cells from TB patients, and three of them (ESAT-6, CFP10 and PPE68) were identified as the major antigens [15]. However, PPE68, was recognized equally well by peripheral blood mononuclear cells (PBMCs) obtained from TB patients and *M. bovis* BCG vaccinated healthy subjects, and its presentation to Th1 cells was HLA-promiscuous [15]. The aim of this study was to confirm the recognition of PPE68 by Th1 cells using antigen-induced T-cell lines from *M. bovis* BCG-vaccinated and HLA-heterogeneous healthy subjects. In addition, the HLA-promiscuous regions of PPE68 were identified by HLA-binding prediction analysis in silico, and the experimental verification was performed using overlapping synthetic peptides of PPE68 and PBMCs from *M. bovis* BCG-vaccinated healthy subjects in IFN-γ assays. Furthermore, the core sequence of the immunodominant peptide was identified by using deletion peptides in IFN-γ assays, and its cross-reactive nature was confirmed by demonstrating the presence in other mycobacterial species by sequence homology search.

## Materials and Methods

### Mycobacterial antigens and peptides

The mycobacterial antigen used in this study was irradiated whole-cell *M. tuberculosis* H37Ra [16]. A total of 220 peptides (25-mers, overlapping by 10 residues) corresponding to 12 proteins of RD1 (Rv3871, PE35, ORF4, PPE68, CFP10, ESAT-6, ORF8, Rv3876, Rv3877, Rv3878, ORF14 and OR15) were designed based on the amino acid sequence deduced from the nucleotide sequence of the predicted genes [17]–[19]. All of the peptides were synthesized by Thermo Hybaid GmBH (Ulm, Germany) using fluonerylmethoxycarbonyl chemistry, and used as described previously [20]. In brief, the stock concentrations (5 mg/ml) of the peptides were prepared in normal saline (0.9%) by vigorous pipetting and frozen at −70°C until used. The working concentrations of each peptide were prepared by further dilution in the tissue culture medium RPM1640. A pool of all 220 peptides (RD1_pool_), and pools of peptides of individual proteins were used in cell cultures to represent RD1 and single proteins, respectively.

### Study subjects

The study subjects were *M. bovis* BCG-vaccinated healthy adults randomly selected from the group of blood donors at the Central Blood Bank, Kuwait. All of the donors were immunized with BCG vaccine following routine immunization protocol applied in Kuwait, i.e. The first immunization was given at 4 ½ years of age, followed by *M. tuberculosis* purified protein derivative (PPD)-skin test at 13 years of age, and a booster immunization with BCG in PPD-skin test negative subjects. At the time of inclusion in the study, all the donors were PPD-skin test positive (>10 mm, as determined with tuberculin PPD RT 23 from the Statens Serum Institute, Copenhagen, Denmark). Written informed consent was obtained from all the subjects to participate in the study, and the study protocol was approved by the Ethics Committee of the Faculty of Medicine, Kuwait University, Kuwait.

### Isolation of peripheral blood mononuclear cells from *M. bovis* BCG-vaccinated healthy subjects and in vitro culture for IFN-γ secretion

Peripheral blood mononuclear cells (PBMCs) were isolated from the buffy coats of each donor by density centrifugation according to standard procedures [20]. In brief, each buffy coat was diluted with warm tissue culture medium (RPMI 1640) at a ratio of 1∶2 and gently mixed. Two volumes of the diluted buffy coat was loaded on top of 1 volume of a Lymphoprep gradient (Pharmacia Biotech., Uppsala, Sweden). After centrifugation, the white ring of PBMCs between the plasma and the Lymphoprep was removed and washed three times with RPMI 1640. The cells were finally suspended in 1 ml complete tissue culture medium [RPMI-1640+10% human AB serum+penicillin (100 U/ml)+streptomycin (100 µg/ml+gentamycin (40 µg/ml)], tested for viability (>98% viable by trypan blue exclusion assay) and counted in a Coulter Counter (Coulter Electronics Ltd., Luton, Bedfordshire, England), as described previously [21].

The antigen-induced secretion of IFN-γ by PBMCs was performed using standard procedures, as described previously [21]–[23]. In brief, PBMCs (2×10^5^ cells/well) suspended in 50 µl complete tissue culture medium were seeded into 96-well tissue culture plates (Nunc Roskilde, Denmark). Antigen/peptide in 50 µl of complete medium was added to the wells in triplicate to a final concentration of 5 µg/ml. The final volume of the culture in the wells was adjusted to 200 µl. The plates were incubated at 37°C in a humidified atmosphere of 5% CO_2_ and 95% air. On day 6, supernatants (100 µl) were collected from antigen-stimulated cultures of PBMCs and were kept frozen at −70°C until assayed for IFN-γ activity. The amount of IFN-γ in the supernatants was quantitated by using Immunotech immunoassay kits (Immunotech SAS, Marseille, France) as specified by the manufacturer. The detection limit of the IFN-γ assay kit was 0.4 IU/ml. Secretion of IFN-γ in response to a given antigen or peptide was considered positive when delta IFN-γ (the IFN-γ concentration in cultures stimulated with antigen/peptide minus the IFN-γ concentration in cultures without antigen/peptide) was ≥3 U/ml [17]. The IFN-γ responses were considered strong with median IFN-γ≥5 U/ml and %positives ≥70%, moderate with median IFN-γ >3 to <5 U/ml and %positives ≥50%, to <70%, and weak with median IFN-γ ≤3 U/ml and %positives <50% [17]. The statistical analysis was performed using Z test to identify significant differences (P<0.05) with respect to % positives in response to peptide pool of PPE68 and the individual peptides.

### HLA typing of PBMCs

Genomic HLA-DR and DQ typing of PBMCs were performed by using sequence specific primers (SSP) in polymerase chain reaction (PCR), as described previously [23]–[25]. HLA-DR “low resolution” kits containing the primers to type for DRB1, DRB3, DRB4 and DRB5 alleles were purchased form Dynal AS (Oslo, Norway) and used according to the manufacturer's instructions. In brief, high molecular weight genomic DNA from PBMCs were isolated by treatment of the cells with proteinase-K and salting out in mini scale. For DR “low resolution” PCR-SSP typing, 21 separate PCR reactions were performed per sample; 17 for assigning DR1 to DRw18 alleles of DRB1 and three for identifying the HLA-DR51, -DR52 and -DR53 super-specificities encoded by DRB3, DRB4 and DRB5, respectively. The genotypes were identified from the size of the amplified products and serologically defined HLA-DR (DR1 to DR18) specificities were determined from the genotypes by following the guidelines provided by Dynal AS.

### Establishing antigen-reactive T-cell lines

Antigen-specific T-cell lines were established from PBMCs by stimulation with the peptide pools of RD1 and PPE68 according to standard procedures [23]–[25]. In brief, 2×10^5^ cells/well were stimulated with 5 µg/ml of peptides in 96 well plates and incubated at 37°C in an atmosphere of 5% CO2 and 95% air for 6 days. Starting from day 6, IL-2 (100 U/well) (Amersham Life Sciences, Amersham, U.K.) was added twice a week until the cell number was sufficient to be transferred to 24 well tissue culture plates (Nunc Roskilde, Denmark). The T-cell lines were maintained in 24 well plates with twice a week addition of IL-2 and tested for antigen reactivity 3–4 days after the last addition of IL-2. The T-cell lines were phenotyped for the expression of CD4 and CD8 molecules using standard procedures [26].

### IFN-γ secretion by T-cell lines

The T-cell lines were tested for antigen-induced IFN-γ secretion in the wells of 96-well tissue culture plates (Nunc, Roskilde, Denmark) in the presence of autologous and allogeneic HLA-typed antigen presenting cells (APCs), as described previously [23], [25]. In brief, adherent cells obtained from irradiated (24 Grays) PBMCs (seeded into the wells of 96-well plates at 1×10^5^ cells/well) were used as APCs. The T-cell lines were added to the wells at a concentration of 5×10^4^ cells/well. Peptides were added in triplicate at a final concentration of 5 µg/ml, and the control wells lacked the peptides. The plates were incubated at 37°C in an atmosphere of 5% CO_2_ and 95% air. After 3 days of incubation, the culture supernatants were collected and assayed for IFN-γ concentrations using immunoassay kits (Coulter/Immunotech, S.A., Marseille, France), as described above for PBMCs. The secretion of IFN-γ in response to a given antigen was considered positive with IFN-γ concentration ≥5 IU/ml [25].

### HLA-DR binding prediction analysis of PPE68 and its peptides

HLA-DR binding prediction analysis of PPE68 and the sequence of each peptide was first performed using the ProPred server (http://www.imtech.res.in/raghava/propred/) at threshold value of 3, as described previously [27]. This server is a useful tool in locating the promiscuous binding regions that can bind to a total of 51 alleles belonging to nine serologically defined HLA-DR molecules [27]–[29]. These HLA-DR molecules are encoded by DRB1 and DRB5 genes including HLA-DR1 (2 alleles), DR3 (7 alleles), DR4 (9 alleles), DR7 (2 alleles), DR8 (6 alleles), DR11 (9 alleles), DR13 (11 alleles), DR15 (3 alleles) and DR51 (2 alleles). The peptides of PPE68 predicted to bind >50% HLA-DR alleles included in the ProPred were considered promiscuous for binding [30].

In addition, ProPred-predicted four HLA-promiscuous and four HLA-non-binder peptides were further analyzed for HLA-DR binding predictions using two other computational prediction methods, i.e. NetMHCIIpan-2.0 [31], and Immuno Epitope Data Base (IEDB) Consensus [32], for binding to 14 alleles, including HLA DRB1*0101, DRB1*0301, DRB1*0401, DRB1*0701, DRB1*1101 and DRB1*1501 supertype alleles that are expected to cover approximately >95% of any given human population [33]. The sequences/peptides predicted to bind >50% alleles of HLA-DR molecules analyzed were considered promiscuous for binding [30].

### Search for sequence identity

The complete PPE68 sequence and the immunodominant and HLA-promiscuous peptide sequence (121-VLTATNFFGINTIPIALTEMDYFIR-145) were searched for identical sequences in various strains of *M. tuberculosis* and mycobacterial species using Protein Basic Local Alignment Search Tool (BLAST), National Center for Biotechnology Information, National Institute of Health, Bethesda, Maryland, USA, using the world wide web (WWW) server.

## Results

### Antigen-specific IFN-γ secretion by human T-cell lines

T-cell lines were established from HLA-heterogeneous donors by stimulating PBMCs with the RD1_pool_ (n = 4 donors, Table 1) and PPE68 (n = 3 donors, Table 2), as the primary antigens *in vitro*. Phenotypic analysis showed that all of these T-cell lines belonged to the CD4+, CD8− subset of T cells. Subsequent testing for antigen-induced IFN-γ secretion demonstrated that all of the four RD1-induced T-cell lines responded to whole-cell *M. tuberculosis* and three of them responded to RD1_pool_ (Table 1). When tested with the peptide pools of individual proteins of RD1, only PPE68 induced positive responses in all of the three T-cell lines responding to RD1_pool_ (Table 1), whereas, only one T-cell line responded to 10 of the 12 ORFs of RD1 (Table 1). The IFN-γ responses of three T-cell lines established against PPE68 were also tested with whole-cell *M. tuberculosis*, PPE68 and peptide pools of some other RD1 proteins, and the results showed that all of these T-cell lines responded to whole-cell *M. tuberculosis* and PPE68, but not to other RD1 proteins (Table 2).

**Table 1:** IFN-γ secretion by RD1-induced T-cell lines from HLA-heterogeneous subjects in response to whole cell *M. tuberculosis*, RD1pool and various ORFs of RD1.

Antigen/Peptides	Concentrations of IFN-γ (IU/ml) in culture supernatants of T-celllines with HLA-type			
	DR7,10,53	DR7,13,52,53	DR11,13,52	DR3,11,52
*M. tuberculosis*	**54**	**57**	**44**	**15**
RD1_pool_	**63**	**37**	**26**	0.7
Rv3871	<0.4	<0.4	1.1	<0.4
PE35	**22**	1.0	1.4	<0.4
ORF4	1.0	<0.4	0.5	<0.4
PPE68	**57**	**44**	**38**	<0.4
CFP10	**40**	0.7	3.0	<0.4
ESAT-6	**71**	2.7	3.0	<0.4
ORF8	**54**	1.0	2.3	<0.4
Rv3876	**69**	1.8	2.6	<0.4
Rv3877	**67**	0.4	1.1	<0.4
Rv3878	**41**	<0.4	1.0	<0.4
ORF14	**28**	<0.4	0.7	<0.4
ORF15	**29**	<0.4	0.4	<0.4

The T-cell lines were established after stimulation of PBMCS with RD1_pool_ and tested for antigen reactivity in IFN-γ assays, as described in the materials and methods. The positive responses (IFN-γ concentration ≥5 U/ml) are given in bold face.

**Table 2:** IFN-γ secretion by PPE68-induced T-cell lines from HLA-heterogeneous subjects in response to whole cell *M. tuberculosis* and various ORFs of RD1.

Antigen/Peptides	Concentrations of IFN-γ (IU/ml) in culture supernatants of T-celllines with HLA-type		
	DR1,11,52	DR2,5,51,52	DR4,7,53
*M. tuberculosis*	**26**	**26**	**30**
PPE68	**27**	**26**	**12**
ORF4	0.4	1.1	1.3
CFP10	1.0	2.1	1.7
ORF8	1.6	0.8	1.5
Rv3877	0.8	2.3	0.9

The T-cell lines were established after stimulation of PBMCS with the peptide pool of PPE68 and tested for antigen reactivity in IFN-γ assays, as described in the materials and methods. The positive responses (IFN-γ ≥5 IU/ml) are given in bold face.

### Identification of immunodominant and HLA-promiscuous peptide(s) of PPE68

To identify the peptides of PPE68 recognized by Th1-type cells, individual peptides of PPE68 were tested with PBMCs from 30 *M. bovis* BCG-vaccinated healthy subjects in IFN-γ assays. The results showed that all of the peptides induced positive responses in a proportion of donors, which ranged from 30% to 70% (Table 3). However, the best responses were observed with peptide P9 (121- VLTATNFFGINTIPIALTEMDYFIR-145), which induced positive responses in 21/30 (70%) subjects. In terms of % positives, the response induced by P9 (121–145) was comparable to the response induced by the full-length PPE68 protein (1–371) with 22/30 (73%) subjects showing positive response (Table 3). Except P9 (21–145), none of the other peptides of PPE68 qualified to be strong stimulator of Th1-type cells, because the IFN-γ responses to them were either moderate (P1, P2, P4, P8, P11, P12, P13, P14, P17, P18, P20, P21) or weak (P3, P5, P6, P7, P10, P15, P16, P19, P22, P23 and P24) (Table 3). These results suggest that, for Th1-type cell-reactivity, only P9 (121–145) was the immunodominant peptide of PPE68.

**Table 3:** Antigen-induced IFN-γ secretion by PBMCs from 30 *M. bovis* BCG-vaccinated healthy subjects and ProPred predictions for PPE68 and its peptides (P1 to P24) to bind 51 HLA-DR alleles.

Peptide	IFN-γ response^a^			HLA-DR binding^b^	
	Median IU/ml	P/T	% positive	P/T	% binding
PPE68 (1–371)	**22**	22/30	**73%**	50/51	**98**
P1 (1-VITMLWHAMPPELNTARLMAGAGPA-25)	3.6	16/30	53%	1/51	2
P2 (16-ARLMAGAGPAPMLAAAAGWQTLSAA-40)	4.3	16/30	53%	6/51	12
P3 (31-AAGWQTLSAALDAQAVELTARLNSL-55)	1.2	10/30	33%	22/51	43
P4 (46-VELTARLNSLGEAWTGGGSDKALAA-70)	3.5	16/30	53%	0/51	0
P5 (61-GGGSDKALAAATPMVVWLQTASTQA-85)	2.3	12/30	40%	35/51	**69**
P6 (76-VWLQTASTQAKTRAMQATAQAAAYT-100)	1.6	13/30	43%	9/51	18
P7 (91-QATAQAAAYTQAMATTPSLPEIAAN-115)	2.6	14/30	47%	0/51	0
P8 (106-TPSLPEIAANHITQAVLTATNFFGI-130)	3.2	16/30	53%	3/51	6
P9 (121-VLTATNFFGINTIPIALTEMDYFIR-145)	**7.9**	21/30	**70%**	33/51	**65**
P10 (136-ALTEMDYFIRMWNQAALAMEVYQAE-160)	2.7	14/30	47%	38/51	**75**
P11 (151-ALAMEVYQAETAVNTLFEKLEPMAS-175)	3.5	15/30	50%	24/51	47
P12 (166-LFEKLEPMASILDPGASQSTTNPIF-190)	3.5	15/30	50%	24/51	47
P13 (181-ASQSTTNPIFGMPSPGSSTPVGQLP-205)	4.6	17/30	57%	23/51	45
P14 (196-GSSTPVGQLPPAATQTLGQLGEMSG-220)	4.6	17/30	57%	2/51	4
P15 (211-TLGQLGEMSGPMQQLTQPLQQVTSL-235)	1.9	13/30	43%	6/51	12
P16 (226-TQPLQQVTSLFSQVGGTGGGNPADE-250)	1.5	12/30	40%	23/51	45
P17 (241-GTGGGNPADEEAAQMGLLGTSPLSN-265)	3.7	17/30	57%	11/51	22
P18 (256-GLLGTSPLSNHPLAGGSGPSAGAGL-280)	3.5	15/30	50%	0/51	0
P19 (271-GSGPSAGAGLLRAESLPGAGGSLTR-295)	1.8	14/30	47%	16/51	31
P20 (286-LPGAGGSLTRTPLMSQLIEKPVAPS-310)	4.2	16/30	53%	19/51	37
P21 (301-QLIEKPVAPSVMPAAAAGSSATGGA-325)	4.1	15/30	50%	29/51	**57**
P22 (316-AAGSSATGGAAPVGAGAMGQGAQSG-340)	0.8	10/30	33%	0/51	0
P23 (331-GAMGQGAQSGGSTRPGLVAPAPLAQ-355)	0.7	9/30	30%	18/51	35
P24 (346-GLVAPAPLAQEREEDDEDDWDEEDDW-371)	1.4	11/30	37%	0/51	0

a IFN-γ responses were evaluated by stimulating PBMCs with the peptides of PPE68 according to procedures described in materials and methods. The strong responses (Median concentration >5 U/ml and %positive≥70%) are given in bold face.

b HLA-DR binding predictions for complete PPE68 sequence and its individual peptides were analyzed using the ProPred server (http://www.imtech.res.in/raghava/propred/). The % binding values suggesting promiscuous HLA-DR binding (binding to >50% HLA-DR alleles) are shown in bold face.

P/T = Number of subjects positive/Number of subjects tested.

In addition to the functional assay for Th1-type cell reactivity, the sequences of PPE68 and its individual peptides were also analyzed for the presence of T-cell epitopes by predicting to bind HLA-DR molecules using the ProPred server. Because the complete PPE68 sequence (1–371) is too large, therefore, binding prediction for all of its peptides to 51 HLA-DR alleles included in ProPred, cannot be presented in a figure or a table. Instead, the summary of HLA-DR binding results are presented in table 3. However, to provide an idea of HLA-DR binding predictions, the prediction results for a small region (106 to 160 covering peptides P8, P9 and P10) to individual HLA-DR alleles, included in ProPred, are shown in fig. 1.

**Figure 1:** ProPred analysis of a part of PPE68 sequence (106–160) using the ProPred server (http://www.imtech.res.in/raghava/propred/) covering three overlapping peptides (P8, P9 and P10) to 51 HLA-DR alleles. The output of ProPred analysis of PPE68 sequence (aa 106–160) for binding to 51 HLA-DR alleles at the default setting (threshold value of 3) is shown in HTML II view. The sequences predicted to bind HLA-DR alleles are underlined. The obligatory anchor (starting) residues are marked in bold.

The overall results of ProPred analysis suggest that PPE68 was a promiscuous HLA-DR binder and T-cell epitopes were scattered throughout the sequence of PPE68 (Table 3). In total, 50/51 (98%) of HLA-DR specificities included in ProPred were predicted to bind PPE68 sequence and 19 of 24 peptides were predicted to be HLA-DR binders (Table 3). However, five peptides of PPE68, i.e. P4, P7, P18, P22 and P24 were not predicted to have T-cell epitopes using ProPred, but the results of IFN-γ assays showed that all of them had Th1 cell-stimulating epitopes and induced moderate (P4) to weak responses (P7, P18, P22, P24) (Table 3). Furthermore, the peptides P5, P9, P10 and P21 were found HLA-promiscuous (Table 3, Fig. 1: data shown for P9 and P10), but only P9 qualified as a strong stimulator, whereas others were weak stimulators of IFN-γ secretion (Table 3). All other peptides were predicted to be non-promiscuous HLA-DR binders, and none of them were strong stimulators of Th1 cells in IFN-γ assays (Table 3).

### Identification of immunodominant and HLA-promiscuous epitope of peptide P9 (121–145)

The immunodominant peptide P9 (121-VLTATNFFGINTIPIALTEMDYFIR-145) of PPE68 is a 25-mer and each amino acid of this sequence contributed in binding to HLA-DR molecules included in ProPred (Fig. 1). It has got six independent sequences (each a 9-mer), which were predicted to bind one (121-VLTATNFFG-129), two (122-LTATNFFGI-130, 135-IALTEMDYF-143 and 137-LTEMDYFIR-145), 16 (128-FGINTIPIA-136) and 28 (127-FFGINTIPI-135) alleles of HLA-DR molecules included in ProPred (Fig. 1). HLA- promiscuous binding of the peptide 121–145 was also suggested by using other prediction programs for binding to HLA-DR alleles, i.e. NetMHCII 2.2, and IEDB Consensus, which predicted to bind 11/14 (79%) and 10/14 (70%) alleles of HLA-DR, respectively. Testing a series of deletion peptides of 121–145 with PBMCs of eight HLA-heterogeneous healthy subjects responding to the full-length peptide showed that the IFN-γ responses (8/8 responders) and HLA-DR binding predictions (33/51, 65%) were fully conserved for the 10-mer sequence 127-FFGINTIPIA-136 (Table 4). However, any further deletion on either side of this core peptide decreased the frequency of positive response as well as the ability to predict binding to HLA-DR alleles by ProPred (Table 4). However, variations were observed in the minimum length of peptides inducing a positive response in various donors, and even 9, 8 and 7-mer peptides, which belonged to the HLA-DR binding region but were not predicted to bind HLA-DR alleles included in the ProPred due to short length (<10 aa), could induce positive responses in PBMCs of six, five and two donors, respectively (Table 4).

**Table 4:** Analysis of peptide 121–145 and its deletions for prediction to bind HLA-DR alleles and secretion of IFN-γ by PBMCs from HLA-DR heterogeneous healthy subjects.

Peptide sequence	HLA-DR binding		Antigen-induced IFN-γ (IU/ml) secretion by PBMCs of donors								P/T^a^
	P/T	% binding	1	2	3	4	5	6	7	8	
**VLTATNFFGINTIPIALTEMDYFIR**	33/51	65	**43**	**5.0**	**28**	**5.0**	**8.0**	**16**	**26**	**9.0**	8/8
ATN**FFGINTIPIALTEMDYFIR**	33/51	65	**41**	**6.0**	**16**	**5.0**	**20**	**22**	**17**	**8.0**	8/8
ATN**FFGINTIPIA**L	33/51	65	**45**	**17**	**19**	**5.0**	**28**	**17**	**12**	**8.0**	8/8
ATN**FFGINTIPI**	38/51	55	**47**	**5.1**	**9.0**	**5.0**	**24**	**14**	**16**	**10**	8/8
**FFGINTIPIA**L	33/51	65	**51**	**5.0**	**19**	**19**	**26**	**16**	**10**	**6.0**	8/8
**FFGINTIPIA**	33/51	65	**50**	**5.0**	**13**	**5.0**	**8.7**	**16**	**15**	**7.0**	8/8
**FGINTIPIA**L	16/51	31	**25**	4.0	**5.0**	**5.0**	**11**	**11**	**13**	**5.0**	7/8
FGINTIPIA	NA^b^	NA	**21**	3.0	1.0	**5.5**	**26**	**17**	**9.0**	**5.0**	6/8
GINTIPIAL	NA	NA	0.5	3.0	4.0	3.5	1.0	3.0	**12**	2.0	1/8
INTIPIAL	NA	NA	0.5	2.0	4.0	1.0	1.0	3.0	**6.0**	4.0	1/8
FFGINTIPI	NA	NA	**57**	2.0	4.0	**5.0**	3.0	**6.0**	**15**	**5.0**	5/8
FFGINTIP	NA	NA	**28**	4.0	**18**	2.5	1.0	**12**	**17**	**5.0**	5/8
FGINTIPI	NA	NA	**28**	2.0	**15**	4.0	3.0	**8.0**	**16**	4.0	4/8
FFGINTI	NA	NA	0.5	2.0	1.0	1.0	3.0	2.0	**9.0**	**7.0**	2/8
FGINTIP	NA	NA	1.0	2.0	4.0	2.5	3.0	1.0	1.8	4.0	0/8

HLA types of donors 1(DR7,17,52,53; DQ2,6), 3(DR11,13,52; DQ7), 4(DR17,52; DQ2) 5(DR1,18,52;DQ4,5), 6(DR14,15,51,52; DQ5,6), 7(DR4,16,51,53;DQ5,8), 8(DR4,17,52,53;DQ2,8).

The regions of peptide 121–145 and its deletions predicted to bind HLA-DR molecules are shown in bold and the anchor sequences are underlined.

a P/T = Number of positive PBMCs donors/Number of donors tested.

b NA = Not applicable. This is because these sequences are <10 aa in length, which is the minimum requirement for ProPred to predict binding of peptide sequences to HLA-DR alleles [27].

A BLAST search for sequence homology with the PPE68 sequence and peptide P9 (121-VLTATNFFGINTIPIALTEMDYFIR-145) in the data base of NCBI showed that PPE68 was 100% conserved in all organisms of *M. tuberculosis* complex, except BCG, and had 75% and 67% identities with PPE proteins of *M. kansasii* and *M. marinum*, respectively, whereas the sequence identities were <40% with PPE proteins of other mycobacteria, including BCG (data not shown). However, the sequence covering the immunodominant and HLA-promiscuous region of peptide 121–145, i.e. 127-FFGINTIPIA-136, was completely identical between proteins encoded by genes of PPE-family proteins present in several mycobacterial strains and species including *M. tuberculosis* complex, i.e. *M. tuberculosis* (>35 strains, including laboratory and drug-susceptible as we all multi-drug resistant clinical isolates), *M. africanum*, *M. bovis*, *M. bovis* BCG and *M. canettii* and non-tuberculous mycobacteria, e.g. *M. avium*, *M. marinum*, *M. ulcerans*, *M. kansasii* and *M. leprae* etc. (Table 5).

**Table 5:** BLAST search data for sequence identity of PPE68 peptide (121–145) in *M. tuberculosis* complex and other pathogenic mycobacteria.

Mycobacterial species	Amino acid sequence
*M. tuberculosis* complex:	
*M. tuberculosis*(>35 species)	VLT*ATN****FF****GINTIPIA*LTEMDYFIR
*M. bovis*	VLT*ATN****FF****GINTIPIA*LTEMDYFIR
*M. bovis*BCG	VLT*ATN****FF****GINTIPIA*LTEMDYFIR
*M. africanum*	VLT*ATN****FF****GINTIPIA*LTEMDYFIR
*M. canettii*	VLT*ATN****FF****GINTIPIA*LTEMDYFIR
Non-tuberculous mycobacteria:	
*M. kansasii*	VLV*ATN****FF****GINTIPIA*LTEADY---
*M. marinum*	VLV*ATN****FF****GINTIPIA*LTEADY---
*M. ulcerans*	VLV*ATN****FF****GINTIPIA*LTEADY---
*M. paraschrofulaceum*	VLV*ATN****FF****GINTIPIA*LTEADY---
*M. abscessus*	VLL*ATN****FF****GINTIPIA*LNEADY-IR
Mycobacterial species JDM601	VLV*ATN****FF****GINTIPIA*LTEADY---
*M. avium*	VLV*ATN****FF****GINTIPIA*LTEADY---
*M. smegmatis*	VLV*ATN****FF****GINTIPIA*LTEADY---
*M. leprae*	FLI*ATN****FF****GINTIPIA**L*NEADYVR-

The 13 aa sequence of PPE68 (aa 124–136) common to all mycobacteria is given in italics and the sequence in each mycobacterial species predicted to bind HLA-DR alleles in this region is underlined. The obligatory anchor (starting) residues for HLA-DR binding are marked in bold.

## Discussion

In this study, PPE68, a major antigenic protein of *M. tuberculosis* was tested for inducing IFN-γ secretion by antigen-induced T-cell lines and identification of immunodominant peptide(s) by testing PBMCs from HLA-heterogeneous *M. bovis* BCG-vaccinated healthy humans. It has previously been shown that, PPE68, although belongs to the group of proteins encoded by *M. tuberculosis*-specific RD1 genomic segment of DNA, was recognized in Th1-cell assays (antigen-induced proliferation and IFN-γ secretion) by PBMCs from *M. tuberculosis*-infected and non-infected *M. bovis* BCG-vaccinated healthy subjects [15], [34]. However, PBMCs are a mixture of various cell types present in the peripheral blood, and therefore the use of PBMCs does not conclusively rule out the recognition of PPE68 by non-T cells or the non-specific mitogenic effect of the protein. Therefore, to confirm that PPE68 was recognized by antigen-specific T cells, antigen-induced T-cell lines from HLA-heterogeneous subjects were established in this study.

Among the antigens used to establish T-cell lines were RD1_pool_ containing peptides of 12 ORFs of RD1, and a pool consisting of the peptides of PPE68 only. Phenotypically, all of the T-cell lines were CD4+, CD8−, confirming the previous observations using similar procedures to establish T-cell lines against other antigens of *M. tuberculosis* [23]–[25]. Furthermore, the T-cell lines from all donors responded to whole cell *M. tuberculosis* suggesting their previous exposure to antigens of *M. tuberculosis* either through infection with *M. tuberculosis* and/or vaccination with *M. bovis* BCG. However, one of the four RD1-induced T-cell line did not respond to RD1pool. This could have been due to the low frequency or absence of RD1-reactive T cells in this cell line. The establishment of a T-cell line from this donor could have been due to the antigen non-specific stimulation of *M. tuberculosis*-reactive T cells by IL-2, as has been shown previously with other antigens [35]. However, all three RD1pool-reactive T-cell lines also responded to PPE68, and only one T cell line responded to nine other RD1 antigens, including ESAT-6 and CFP10 (Table 1). All of the three T-cell lines established against PPE68 responded to this antigen only (Table 2), which suggests that the responses to PPE68 were antigen-specific and not due to the activation of non-specific T cells.

The positive responses of PBMCs from healthy subjects to ESAT-6/CFP10 have been considered as indication of prior infection of donors with *M. tuberculosis* [36]–[38]. Thus, the positive responses of T-cell lines to PPE68, but not to other RD1 antigens, suggest that these donors were not infected with *M. tuberculosis*, and therefore, the positive responses to PPE68 could have been due to vaccination with BCG and/or exposure to environmental mycobacteria, as suggested previously for other crossreactive antigens of *M. tuberculosis*, e.g. MPT63, MPB70 and MPT83 etc. [29], [39].

To identify immunodominant epitope(s) in PPE68, two approaches were used in this study. First PBMCs from HLA-heterogeneous subjects were tested with 24 overlapping peptides covering the sequence of PPE68. A similar approach has previously been used to identify the immunodominant epitopes of other major antigenic proteins of *M. tuberculosis* [40]–[42]. The results showed that all of the peptides of PPE68 induced positive responses in a proportion of donors, but, the best responses were observed with peptide P9 (121- VLTATNFFGINTIPIALTEMDYFIR-145). Although, T-cell epitopes were present throughout the sequence of PPE68, the percent positive response induced by P9 (121–145) was comparable to the percent positive response induced by the peptide pool of full-length PPE68 protein (1–371) (P>0.05, by Z test). This feature seems to be unique to this peptide, because none of the single peptides of other mycobacterial proteins have shown similar positivity in human Th1-cell assays, as full-length proteins [29], [39]–[44].

In addition to Th1-cell reactivity, the sequences of PPE68 and its individual peptides were analyzed for the presence of T-cell epitopes using the ProPred server, which predicts binding to molecules encoded by 51 HLA-DR alleles [27]. The ProPred analysis has previously been shown to identify immunodominant antigens and peptides of several *M. tuberculosis* proteins [28]–[30], [39], [40]. The overall results of ProPred analysis suggest that PPE68 was a promiscuous HLA-DR binder (Table 3). The analysis of individual peptide sequences by ProPred suggested that 19 of 24 peptides were predicted to be HLA-DR binders (Table 3). However, five peptides of PPE68, i.e. P4, P7, P18, P22 and P24 were not predicted to have T-cell epitopes by ProPred analysis, but the results of IFN-γ assays showed that all of them had T-cell epitopes and induced moderate (P4 and P18) to weak responses (P7, P22, P24) (Table 3). The discrepancy between the HLA-DR binding and the functional assay could be due to the reason that ProPred, although includes the binding prediction for a large number of HLA-DR molecules, does not include all HLA-DR specificities [27]. Alternatively, ProPred is not 100% accurate to predict the binding [28]–[30], [39], [40]. Therefore, the five non-binding and four promiscuous peptides of PPE68 were further evaluated for binding predictions using two additional servers, i.e. NetMHCII 2.2 and IEDB Consensus, which are suggested to have similar overall performance as ProPred, but differ in their binding predictions to individual HLA-DR alleles [45], [46]. The results suggested that all of the five peptides suggested to be non-binders by ProPred were binders by NetMHCII 2.2 and three of them were also predicted to bind HLA-DR alleles by IEDB Consensus method (Table 6). Furthermore, among four peptides suggested to be promiscuous binders by ProPred, only three peptides (P5, P9 and P10) were promiscuous binders by other two methods. Importantly P9 and P10 were suggested to be promiscuous binders by all three methods but only P9 was immunodominant in IFN-γ assays (Table 6). This could be due to the reason that binding of peptides to HLA-DR molecules, although essential for recognition by Th1 cells, is not sufficient for Th1-cell recognition, because the later requires the existence of cells with epitope-specific T-cell receptors, which may be lacking in some individuals.

**Table 6:** Comparison of binding predictions of selected peptides of PPE68 to HLA-DR alleles using various computational methods and IFN-γ responses of PBMCs from 30 healthy subjects.

Peptide	Binding to HLA-DR alleles predicted by^a^			Subjects responding in IFN-γ assays^b^
	ProPred	NetMHCII 2.0	IEDB Consensus	
P4 (46–70)	0/51 (0%)	4/14 (29%)	1/14 (7%)	16/30 (53%)
P7 (91–1155)	0/51 (0%)	6/14 (43%)	3/14 (21%)	14/30 (47%)
P18 (256–280)	0/51 (0%)	4/14 (29%)	0/14 (0%)	15/30 (50%)
P22 (316–340)	0/51 (0%)	1/14 (7%)	0/14 (0%)	10/30 (33%)
P24 (346–371)	0/51 (0%)	2/14 (14%)	1/14 (7%)	11/30 (37%)
P5 (61–85)	**35/51 (69%)**	**11/14 (79%)**	7/14 (50%)	12/30 (40%)
P9 (121–145)	**33/51 (65%)**	**11/14 (79%)**	**10/14 (71%)**	**21/30 (70%)**
P10 (136–160)	**38/51 (75%)**	**12/14 (86%)**	**11/14 (79%)**	14/30 (47%)
P21 (301–325)	**29/51 (57%)**	3/14 (21%)	3/14 (21%)	15/30(50%)

a The results are shown as number of HLA-DR molecules predicted to bind/number of HLA-DR molecules tested for binding to a given peptide and the percentages are given in brackets.

b The results are given as the number of subjects positive/the number of subjects tested with each peptide and the percentages of positi9ve responders are given in brackets.

The %binding values suggesting promiscuous HLA-DR binding (binding to >50% HLA-DR alleles) and the strong responses (Median IFN-γ concentration >5 U/ml and %positive ≥70%) are given in bold face.

The immunodominant peptide P9 (121-VLTATNFFGINTIPIALTEMDYFIR-145) of PPE68 is a 25-mer and each amino acid of this sequence contributes in binding to HLA-DR molecules included in ProPred (Fig. 1). However, a 10 aa sequence, i.e. 127-FFGINTIPIA-136 retained the full capacity to stimulate Th1 cells and to bind HLA-DR molecules by ProPred (Table 4). The same sequence also retained its promiscuous character for binding to HLA-DR alleles, when analyzed by NetMHCII 2.2 and IEDB Consensus methods (data not shown). Thus, both functional as well as methods for T-cell epitope prediction unanimously confirm immunodominant nature of the sequence 127-FFGINTIPIA-136 for recognition by CD4+ Th1 cells.

A search for sequence homology with the peptide P9 sequence (121-VLTATNFFGINTIPIALTEMDYFIR-145) in the data base of National Centre for Biotechnology Information, USA, using Basic Local Alignment Search Tool (BLAST) for comparing protein sequences, showed that a 13 aa stretch, i.e. 124-ATNFFGINTIPIA-136), was completely identical between proteins encoded by genes of other PPE-family proteins present in various mycobacterial strains and species, e.g. *M. tuberculosis*, *M. bovis*, *M. bovis* BCG, *M. avium*, *M. marinum*, *M. ulcerans* and *M. leprae* etc. (Table 5). These results suggest that the core region of the immunodominant peptide of PPE68, i.e. 127-FFGINTIPIA-136, is present in several pathogenic mycobacteria. Furthermore, the full length peptide 121–145 as well as peptide 127–136 were also suggested to possess CD8+ cytotoxic T cell epitopes using nHLAPred/Compred [47] and ProPred-I [48] (Table 7). Since the involvement of both CD4+ and CD8+ T cells is suggested for optimal protection against mycobacterial disease [49], [50], the use of crossreactive peptide 121-VLTATNFFGINTIPIALTEMDYFIR-145 of PPE68 may be useful as a peptide-based vaccine against TB and other mycobacterial diseases.

**Table 7:** Binding predictions forPPE68peptides 121–145, 124–137 and 127–136 to HLA-class I alleles using the prediction methods nHLAPred/Compred and ProPred-I.

Peptide	Binding to HLA-class I alleles predicted by^a^	
	nHLAPred/Compred	ProPred-I
121-VLTATNFFGINTIPIALTEMDYFIR-145	25/67 (37%)	41/47(87%)
124-ATNFFGINTIPIAL-137	15/67(22%)	26/47(55%)
127-FFGINTIPIA-136	4/67(6%)	15/47(32%)

a The results are shown as no. of HLA-class I molecules predicted to bind/number of HLA-class I molecules tested for binding to a given peptide and the binding percentages are given in brackets.
